# Three-Dimensional Gait Analysis and sEMG Measures for Robotic-Assisted Gait Training in Subacute Stroke: A Randomized Controlled Trial

**DOI:** 10.1155/2023/7563802

**Published:** 2023-04-11

**Authors:** Huihuang Zhang, Xiang Li, Yichen Gong, Jianing Wu, Jianer Chen, Weihai Chen, Zhongcai Pei, Wanying Zhang, Lei Dai, Xinxin Shu, Cheng Shen

**Affiliations:** ^1^The Third Clinical Medical College, Zhejiang Chinese Medical University, 310053 Hangzhou, Zhejiang, China; ^2^Department of Center for Rehabilitation Assessment and Therapy, Zhejiang Rehabilitation Medical Center, 310053 Hangzhou, Zhejiang, China; ^3^The Third Affiliated Hospital of Zhejiang Chinese Medical University, 310013 Hangzhou, Zhejiang, China; ^4^Neurorehabilitation Department, Zhejiang Rehabilitation Medical Center, 310053 Hangzhou, Zhejiang, China; ^5^Department of Hangzhou Innovation Institute, Beihang University, 310053 Hangzhou, Zhejiang, China

## Abstract

**Background:**

The efficacy of robotic-assisted gait training (RAGT) should be considered versatilely; among which, gait assessment is one of the most important measures; observational gait assessment is the most commonly used method in clinical practice, but it has certain limitations due to the deviation of subjectivity; instrumental assessments such as three-dimensional gait analysis (3DGA) and surface electromyography (sEMG) can be used to obtain gait data and muscle activation during walking in stroke patients with hemiplegia, so as to better evaluate the rehabilitation effect of RAGT.

**Objective:**

This single-blind randomized controlled trial is aimed at analyzing the impact of RAGT on the 3DGA parameters and muscle activation in patients with subacute stroke and evaluating the clinical effect of improving walking function of RAGT.

**Methods:**

This randomized controlled trial evaluated the improvement of 4-week RAGT on patients with subacute stroke by 3DGA and surface electromyography (sEMG), combined with clinical scales: experimental group (*n* = 18, 20 sessions of RAGT) or control group (*n* = 16, 20 sessions of conventional gait training). Gait performance was evaluated by the 3DGA, and clinical evaluations based on Fugl-Meyer assessment for lower extremity (FMA-LE), functional ambulation category (FAC), and 6-minute walk test (6MWT) were used. Of these patients, 30 patients underwent sEMG measurement synchronized with 3DGA; the cocontraction index in swing phase of the knee and ankle of the affected side was calculated.

**Results:**

After 4 weeks of intervention, intragroup comparison showed that walking speed, temporal symmetry, bilateral stride length, range of motion (ROM) of the bilateral hip, flexion angle of the affected knee, ROM of the affected ankle, FMA-LE, FAC, and 6MWT in the experimental group were significantly improved (*p* < 0.05), and in the control group, significant improvements were observed in walking speed, temporal symmetry, stride length of the affected side, ROM of the affected hip, FMA-LE, FAC, and 6MWT (*p* < 0.05). Intergroup comparison showed that the experimental group significantly outperformed the control group in walking speed, temporal symmetry of the spatiotemporal parameters, ROM of the affected hip and peak flexion of the knee in the kinematic parameters, and the FMA-LE and FAC in the clinical scale (*p* < 0.05). In patients evaluated by sEMG, the experimental group showed a noticeable improvement in the cocontraction index of the knee (*p* = 0.042), while no significant improvement was observed in the control group (*p* = 0.196), and the experimental group was better than the control group (*p* = 0.020). No noticeable changes were observed in the cocontraction index of the ankle in both groups (*p* > 0.05).

**Conclusions:**

Compared with conventional gait training, RAGT successfully improved part of the spatiotemporal parameters of patients and optimized the motion of the affected lower limb joints and muscle activation patterns during walking, which is crucial for further rehabilitation of walking ability in patients with subacute stroke. This trial is registered with ChiCTR2200066402.

## 1. Introduction

Stroke is one of the most common causes of disability in the world [1]. The impairments left after stroke such as motor disorders and cognitive impairments will affect the quality of life of patients for a long time.

Walking is considered the foundation of autonomous mobility; thus, it is necessary to make gait recovery as a primary goal in stroke rehabilitation [2]. The gait function of stroke patients is characterized by the asymmetry of parameters which were used to describe the gait pattern [3, 4]. Therefore, gait rehabilitation should focus on rectifying the coordination disorder and require a large amount of repetitive training [5]. Conventional gait rehabilitation is usually labor intensive, which may require two or three therapists to manually guide the affected limb to follow the correct trajectory [6], placing a significant physical burden on the physiotherapist. Robotic-assisted rehabilitation is a burgeoning field that holds promise as an effective program for automated training. There are two main categories of robotic devices used for body functional rehabilitation: exoskeletons and end-effector robots [7]. In the field of rehabilitation of nervous system diseases (such as stroke), lower extremity exoskeletons are the most commonly used [8]. The lower extremity exoskeletons can be further divided into treadmill-based robots with body weight support (BWS) system and overground robots, which can be worn on the lower extremities of the subjects and directly generate torque on one or more joints to drive them to walk overground [9].

At present, lower limb exoskeletons could satisfy most of the gait rehabilitation needs of stroke patients: improve the patients' balance function in standing position (assisted and unassisted); increase the range of motion (ROM) of the joints (especially hip and knee joints); strengthen the patients' muscle strength during walking; the movement pattern of patients was improved and abnormal gait was rectified [10]. Lower extremity exoskeletons can improve musculoskeletal and neuromuscular performance and may also contribute to neuroplasticity [11]. These mechanisms are crucial for the recovery of motor control, and thus, lower extremity exoskeletons can be considered as a rehabilitation therapy that could produce more complex and controllable multisensory stimulation for patients and alter the plasticity of neural connections through motor training [12]. Compared with conventional gait training, lower extremity exoskeletons could represent an innovative rehabilitation program because they provide high-repetition gait training, even for patients who are unable to maintain an upright posture [13], induce multisensory motor control in patients with severely impaired walking function, and provide the patient with proprioception input during limb loading, which is associated with visual-motion control in order to correctly navigate the motor setting [7]. In clinical practice, robotic-assisted gait training (RAGT) for stroke patients can be performed using lower extremity exoskeletons. The lower extremity exoskeletons for gait rehabilitation conduct walking training by guiding the lower extremity movement of patients through preprogrammed gait patterns. The preprogrammed gait pattern is similar to physiological gait, which includes gait cycle timing, interlimb and interjoint coordination, appropriate limb loading, and afferent signals.

For stroke patients, lower extremity exoskeletons have been proven to effectively help them improve their walking ability, rectify abnormal gait, promote motor function recovery, and improve balance function [14, 15]. That robotic training has significant advantages over conventional rehabilitation training in the rehabilitation treatment of stroke patients with hemiplegia.

As a new tool of rehabilitation therapy, the clinical effect of lower extremity rehabilitation robots needs to be considered and evaluated versatilely. Gait assessment is one of the most important measures to determine therapeutic schedules and evaluate the rehabilitation effects. Observational gait assessment is the most commonly used method in clinical practice, but it has certain limitations due to the deviation of subjectivity [16]. In recent years, the instrumental assessments that can be used during walking have aroused people's concern. In clinical practice, the three-dimensional gait analysis (3DGA) system can be used to accurately detect the walking function of stroke patients [17]. 3DGA mainly includes two systems: motion data acquisition and analysis. The motion data acquisition system includes reflective markers and 3D cameras, which can accurately measure the gait data of the subject by capturing the motion trajectories of the reflective markers attached to the subject. The analysis system includes a motion analysis host and various analysis software. For example, modeling software is needed to build a human body model and analyze it. For gait analysis, gait analysis software is required. Sometimes, three-dimensional force-measuring platforms are needed to measure the ground reaction forces. Previous studies [18–20] have shown that 3DGA is effective in assessing the walking function after stroke.

When human muscles contract, they will generate corresponding electrical activity. Electrophysiological assessment can be used to objectively assess the relevant physiological status of the patients. Surface electromyography (sEMG) is a noninvasive, convenient, and low-cost method to record the activity intensity and activation pattern of muscles in subjects, and this technology has the potential to be widely used in clinical settings. The commonly used metrics of sEMG are divided into time domain metrics and frequency domain metrics. Time domain metrics include integrated electromyography (iEMG), root mean square (RMS), and average electromyography (AEMG), and frequency domain metrics include mean power frequency (MPF) and median frequency (MF). When voluntary muscle contractions are detected, sEMG signals could tell us the muscle activity of the patients during gait, identifying the abnormal activation patterns of muscles, which may affect walking function [21]. In addition, abnormal cocontraction is considered to be one of the important factors limiting the function recovery of stroke patients [22]. Cocontraction refers to the simultaneous action of active and antagonistic muscles on the same joint, which is a mechanism involved in the regulation of joint activity and postural stability [23]. The use of sEMG metrics to calculate the cocontraction rate (CR) of lower extremity joints in stroke patients during walking [24] can accurately and effectively evaluate the gait function level of patients. Studies of sEMG have shown that the cocontraction of knee joint muscles on the affected side of stroke patients increases during the double support phase and the swing phase [25]. Yuan et al. [26] conducted sEMG detection of rectus femoris and biceps femoris muscle in stroke patients and also found that, in stance phase, the cocontraction of the knee joint of the affected side was higher than that of the unaffected side. These results suggest that stroke patients could take weakening the cocontraction of antagonistic muscles as one of the rehabilitation goals.

The purpose of this study is to analyze the impact of RAGT on the clinical walking ability indicators, spatiotemporal parameters, kinematic parameters, and indicators of sEMG in patients with subacute stroke by comparison between RAGT and conventional gait training and evaluate the clinical effect of improving walking function of RAGT.

## 2. Methods

This is a prospective, single-blind, randomized, controlled study with 2 parallel groups. This study was conducted with approval from the Ethics Committee of the Zhejiang Rehabilitation Medical Center (ZKLL20210701). This study was conducted in accordance with the declaration of Helsinki. Written informed consent was obtained from all participants.

### 2.1. Participants

All participants in the study were recruited from Zhejiang Rehabilitation Medical Center. The inclusion criteria for this study were as follows: hemiplegia after first stroke, age > 18 years, less than 6 months since onset, lover extremity modified Ashworth scale (MAS) ≤ 2 [27], walking at least 15 m without assist, and ability to understand and follow instructions. Patients with extreme osteoporosis, unstable fracture, or excessive spasticity were excluded from the study. Other exclusion criteria were severe cognitive impairment, speech impairment, unable to cooperate with training, and deteriorating condition.

### 2.2. Study Protocol

Patients in this study were allocated equally to either the experimental group (RAGT) or the control group (conventional gait training) according to random number table. All participants received 20 sessions, once a day with 30 minutes, 5 days a week for 4 weeks (the flowchart of the study is shown in Figure 1).

### 2.3. Interventions

For the experimental group, patients received RAGT on a lower extremity rehabilitation robot (MANBUZHEKANGFU, Tianjin, China, model: GR-A1) with body weight support (BWS) system (Figure 2); it has linear actuation on the hip and knee joints. During training, the patient wore a harness connected to the robotic system to provide body weight support, and then, the machine drove the patient to walk on the treadmill, simulating a complete physiological gait cycle. Spring elastic bands were used to help to hold the patients' ankle joint in place and prevent foot drop. During training, the robotic lower limb joints were adjusted to the maximum range set by the device. For the first session, the walking speed of the robot was adjusted on 0.5 m/s, and the 50% body weight support was provided. In the next sessions, the walking speed was progressively increased to 2.5 m/s, and degree of BWS was decreased to 0% progressively.

Patients in the control group received conventional gait training. Each patient was instructed to walk on a flat indoor corridor without interruption until they reached an intensity corresponding to a score of 4 on the Borg fatigue index [28]. When this intensity was reached, the patient was allowed to sit in a chair and rest; after an appropriate rest period, the training would start again following the previously stated steps until the end of the training. The entire training session was conducted under the supervision and protection of therapists to prevent adverse events such as falls.

### 2.4. Data Acquisition and Processing

3DGA data: 4 pieces of AMTI force measuring tables (Advanced Mechanical Technology, Inc. USA) and 6-camera VICON (Vicon Motion System) system were used to obtain the spatiotemporal parameters and kinematic data of the patients' gait. The patients were required to wear the same pair of shoes while data were collected before and after treatment. For the test, the VICON PlugInGait LowerBody Ai model (Figure 3) with 16 reflective markers was used to obtain joint movements of the lower extremities; the patients were instructed to walk in the test area with a comfortable gait speed.

sEMG signals: bioelectrical signals generated during lower extremity muscle activity were collected with surface electromyography device (Noraxon, Scottsdale, AZ, USA) at 1500 Hz sampling frequency and synchronized with the VICON motion system during 3D gait assessment. The selected muscles were tibialis anterior, gastrocnemius lateral, rectus femoris, and biceps femoris (Figure 4). The Surface ElectroMyoGraphy for the Noninvasive Assessment of Muscles (SENIAM) was used to locate the sEMG electrodes to minimize signal crosstalk. Before electrode placement, the skin surface of the tested muscles was cleaned with ethanol for disinfection to reduce the impedance. Two Ag/AgCl electrodes were attached to the muscle belly of the tested muscles and arranged along the direction of the muscle fiber. The center distance between the two electrodes was 1 cm.

### 2.5. Outcome Measures

#### 2.5.1. Primary Outcome Measures

3DGA: each patient underwent 3D gait assessment at baseline (before treatment) and after 20 sessions of RAGT over a 4-week period, all performed by the same therapist. Vicon Nexus 2.6.1 software was used to preprocess the collected gait data, and the gait cycle of the raw data was divided (one gait cycle was defined as one heel strike to the next heel strike on the same side), and 3-5 gait cycles were retained for each segment of data (Figure 5). Then, the Vicon Polygon 4.4.3 software was used to analyze the processed gait data, and the data were time normalized according to the percentage of a complete gait cycle (0-100%), and the spatiotemporal parameters (walking speed, stride length, and temporal symmetry index) were recorded. Temporal symmetry index: we took the ratio of the single support time of the unaffected side and the affected side of the patient as the symmetry index (the smaller value was taken as the molecule). Kinematic parameters (ROM of the hip joint in the sagittal plane, peak flexion angle in the swing phase of the knee joint, and ROM of the ankle joint in the sagittal plane) were recorded.

Surface electromyography: we used the Noraxon MR (Version 3.18, USA) software to synchronize the collected EMG signals with the gait cycle of 3D gait data (Figure 6), then performed full-wave rectification on the original EMG signals, and took the absolute value of the signal amplitude; then, a band-stop filter with a 49.5-50.5 Hz stop-band was used to reduce power frequency interference, and a band-pass filter was used too; the pass-band frequency was 30-350 Hz. The processed data was also normalized according to the percentage of a complete gait cycle (0-100%) and divided into stance phase and swing phase. The average EMG (AEMG) amplitude of the affected lower limb in swing phase was taken to calculate the cocontraction index (CCI) in swing phase of knee flexion and ankle dorsiflexion. The formula was as follows:

(1) $$\begin{array}{c} \text{CCI}=\frac{\text{antagonistic muscle AEMG}}{\text{antagonistic muscle AEMG}+\text{agonisitc muscle AEMG}}. \end{array}$$

#### 2.5.2. Clinical Outcomes

Clinical assessments included (1) functional ambulation category (FAC) [29], which consists of a 6-level scale that assesses independent walking function; (2) Fugl-Meyer assessment for lower extremity (FMA-LE) [30], which mainly reflects the active activity of the affected lower extremity, including reflexes, cooperative movement of extension and flexor muscles, coordination ability, and speed, with a total score of 34; and (3) 6-minute walk test (6MWT) [31]: the distance of overground walking for 6 minutes was recorded, and the endurance was evaluated.

## 3. Statistical Analysis

Statistical analyses were performed with the Statistical Packages for Social Sciences (SPSS) (SPSS 25.0, IBM, Chicago, IL, USA), and normally distributed data were expressed as the mean (SD); nonnormal data were expressed as the median (interquartile range). The Shapiro-Wilk test was used to test the normal distribution. Two-sample *t*-test and nonparametric Mann–Whitney test were used to compare two groups of continuous variables. Fisher's precision probability test was used for enumeration data. For the test results, *α* = 0.05 was used as the test level. If *p* < 0.05, the difference was statistically significant.

## 4. Results

38 patients participated in this study, with 4 patients dropped out for personal reasons and 34 patients completed the entire training, including 18 patients of the experimental group and 16 patients of the control group; as for sEMG data, the devices of sEMG were damaged while 1 patient experienced 3D gait capture; and 3 patients had skin allergies to the Ag/AgCl electrodes, if the electrodes were placed, which may cause skins to ulcerate; therefore, we collected sEMG data from 30 patients, including 17 in the experimental group and 13 in the control group. All the patients were evaluated at *T*0 and *T*1. The demographic characteristics of the participants who completed the protocol are shown in Tables 1 and 2; there were no significant differences in age, sex, stroke duration, affected side (left/right), and modified Ashworth scale (MAS) between the two groups and the baseline assessments (FMA-LE, FAC, 6MWT, gait parameters, and sEMG indicators) too. No adverse events were observed during or after training.

### 4.1. Intragroup Comparison

The results of intragroup comparison are showed in Table 3.

In terms of spatiotemporal parameters, after 4-week interventions, walking speed (*p* < 0.001), stride length of the affected side (*p* < 0.001) and the unaffected side (*p* < 0.001), and temporal symmetry index (*p* < 0.001) of the experimental group were significantly improved from baseline; as for the control group, noticeable improvements were found in walking speed (*p* = 0.040), stride length of the affected side (*p* = 0.010), and temporal symmetry index (*p* = 0.021), while there was no statistical difference in stride length of the unaffected side (*p* = 0.393).

The results of kinematics showed that the ROM of the bilateral hip joint (*p* < 0.001 in the affected side, *p* = 0.018 in the unaffected side), flexion angle of the affected knee joint (*p* = 0.001), and ROM of the affected ankle joint (*p* < 0.001) were noticeably improved in the experimental group, while no significant improvement was observed in the flexion angle of the unaffected knee joint (*p* = 0.983) and the ROM of the unaffected ankle joint (*p* = 0.054); and in the control group, the ROM of the affected hip joint (*p* = 0.010) and the ROM of the affected ankle joint (*p* = 0.023) were significantly improved, while no statistical differences were observed in the ROM of the unaffected hip joint (*p* = 0.276), the flexion angle of the bilateral knee joint (*p* = 0.068 in the affected side, *p* = 0.908 in the unaffected side), and the ROM of the unaffected ankle joint (*p* = 0.793) (Figures 7–9).

As for clinical outcomes, compared with their baselines, the experimental group showed significant improvements in FMA-LE (*p* < 0.001), FAC (*p* = 0.001), and 6MWT (*p* < 0.001) after intervention, and FMA-LE (*p* = 0.008), FAC (*p* = 0.002), and 6MWT (*p* = 0.002) were noticeably enhanced in the control group too.

### 4.2. Intergroup Comparison

The results of intergroup comparison are showed in Table 4.

In spatiotemporal parameters of the experimental group, walking speed increased significantly compared with that of the control group (*p* = 0.025), and the improvement of symmetry index was also significantly higher than that in the control group (*p* = 0.004), but the change of stride length on both the affected side (*p* = 0.058) and the unaffected side (*p* = 0.058) was not statistically significant compared with that in the control group.

Intergroup results of kinematics: in terms of the affected side, the experimental group had higher improvement in ROM of the affected hip joint (*p* = 0.032) and flexion angle of the affected knee joint (*p* = 0.001) than the control group; no significant difference was observed in the improvement of the affected ankle (*p* = 0.586) in the experimental group compared with the control group. In terms of the unaffected side, no statistical differences were observed in the unaffected hip joint (*p* = 0.918), knee joint (*p* = 0.065), and ankle joint (*p* = 0.159) in the experimental group when compared with the control group (Figures 7–9).

And results of clinical outcomes showed us that the improvements of FMA-LE (*p* = 0.008) and FAC (*p* = 0.002) in the experimental group were better than those in the control group, but the change of 6MWT (*p* = 0.448) showed no statistical difference between the two groups.

### 4.3. sEMG Cocontraction Index (CCI)

Due to damage to the device of sEMG and skin allergies of patients, we collected sEMG data from 30 patients, including 17 in the experimental group and 13 in the control group, to calculate the cocontraction index of the knee and ankle of the affected lower extremity.

Intragroup results of knee joint (Table 3) showed us that the CCI of the knee in the experimental group was remarkably changed after intervention (*p* = 0.042), while that in the control group was not significantly changed (*p* = 0.196), and intergroup comparison (Table 4) showed that the experimental group was better than the control group (*p* = 0.020). In terms of ankle CCI, we found no significant differences in either the experimental group (*p* = 0.691) or the control group (*p* = 0.753) after intragroup comparison (Table 3); intergroup results (Table 4) also showed that there was no remarkable difference between two groups (*p* = 0.983) (Figure 10).

## 5. Discussion

Rehabilitation robots integrate a variety of technologies and show the characteristics of interdisciplinary areas, mainly used to provide locomotor assistance and rehabilitation treatment for the aged and patients with limb motor dysfunction [32]; even with plentiful advantages, the clinical efficacy of rehabilitation robots still needs more researches and verification. This study is aimed at analyzing the impacts of RAGT on 3DGA parameters and muscle activities of patients with stroke and at examining its clinical efficacy in improving the locomotor function. The results of this study showed that either RAGT with lower extremity robot or conventional gait training could significantly improve the walking dysfunction of walking ability after stroke. However, the patients that received RAGT experienced more improvement in 3D gait parameters and muscle activation pattern than the patients that received conventional gait training. Therefore, RAGT may be an effective solution for the treatment of walking dysfunction after stroke. Besides, rehabilitation robots are generally safe, do not pose risks to patients, and greatly reduce the pressure of rehabilitation therapists.

Gait of poststroke usually presents an asymmetrical pattern, with decreased motor function and shortened stride length of the affected side. At the same time, the stance time of the affected side is relatively shortened, while that of the unaffected side is prolonged. Such changes in spatiotemporal parameters lead to the decline of balance function and affect the walking speed of stroke patients [33]. Walking speed is one of the important parameters to evaluate the functional status after stroke, and the improvement of walking speed is commonly directly related to the patients' daily life quality. In the experimental group of this study, the walking speed significantly improved. We believe that the lower extremity robot can help patients fully initiate joint flexion and lower limb swing, which is conducive to the improvement of walking speed and cadence. The minimum clinically important difference (MCID) in walking speed among subacute stroke patients was 0.16 m/s [34]. In this study, the walking speed of the experimental group was improved to 0.26 m/s, higher than the MCID previously obtained. But in the results of 6MWT, RAGT showed no statistical difference compared with conventional gait training; it may on account of that in 3D gait measurement, patients of two groups with only a short time of walk, while during the 6-minute long walk, patients may have differences in performance due to endurance and compensatory ways. We believe that 6MWT involves many aspects, including endurance, walking function, and balance function; meanwhile, the length of track layout had different effects on different patients [35], and the benefits of enhancement of walking speed may be diluted by subsequent fatigue [36].

In terms of symmetry, the improvement of the experimental group was better than that of the control group, which may be because the BWS system of the robot can reduce the load on the affected lower extremity of the patient, so that the patient could shift the center of gravity to the affected side more easily and walk symmetrically on the robot. The change of symmetry represents the change of patients' ability to control their gait patterns. Jeannine et al. [37] studied the change of pusher behavior in patients with subacute stroke by RAGT and proved the effectiveness of RAGT in reducing pusher behavior in patients with stroke. Pusher behavior refers to the condition that hemiplegia patients after stroke lean to the affected side and resist any correction that makes their body move to the midline or the unaffected side [38], which is closely related to the gait asymmetry of stroke patients. A cross-sectional study [39] found that the gait quality of stroke patients measured by spatial and temporal symmetry appears to deteriorate continuously over time, so improvement of temporal symmetry in stroke patients is an important aspect to promote gait recovery.

The improvement in kinematics of the experimental group was better than that of the control group, which was consistent with our original expectation. The launch of physiological gait refers to the flexion of the hip at the initial stage of the swing phase to accelerate the forward swing of the lower limb [40]. RAGT can input this gait pattern for patients in a highly repetitive mode to drive the patients' lower limb joints to move in the right direction, which is an important part in the motor relearning of patients after stroke. Improvements in ROM of the hip led to more adequate start of gait, and improvements in ROM of the unaffected hip also indicated that RAGT corrected abnormal gait. In terms of the knee, knee flexion in the experimental group was remarkably improved compared with that in the control group after training, and the cocontraction index of the knee also showed a significant improvement, which may be related to the different levels of knee's active movement in two groups during training. In the gait pattern of healthy people, the activation of lower limb muscles is coordinated and rhythmic to ensure the coordination between limbs. In the process of gait in stroke patients, the affected hip needs to increase flexion to cope with foot drop. This enhanced activation of flexor muscle of the hip commonly leads to increased reflex excitability of the rectus femoris [41], abnormal cocontraction degree of the muscles around the knee, and reduced flexion angle of the knee during swing phase. Patients who received RAGT were able to carry out sufficient activities with the assistance of the robot, while in the conventional gait training due to the lack of robot guidance may rely more on the compensatory activities of the trunk and pelvis to ensure the clearance of the foot. Alingh et al. [42] analyzed the results of 32 subacute participants; at 4-month follow-up, the knee flexion angle of the RAGT group showed significant improvement (compared with baseline), while that of the control group did not (compared with baseline), which is similar to the results of our study. In addition, there was no significant difference in ROM of the ankle between two groups after training, and no statistical difference was found in the analysis of cocontraction in sEMG too. The possible explanation for this is that the correct control of ankle activity is controlled by multiple factors such as muscle strength, appropriate muscle activity, sufficient muscle cocontraction, and sensory and visual abilities [43]. The lower limb robot used in this study is not equipped with ankle actuator, but only prevent foot drop through spring elastic bands; the active participation of the ankle was insufficient, so the RAGT did not show significant advantage in improving ankle joint.

In conclusion, we believe that the improvement of RAGT for patients with subacute stroke is more focused on the performance of gait pattern, such as correcting postural asymmetry, guiding the affected joints to move in the right directions during walking, and rectifying abnormal muscle activation patterns. The significant differences in spatiotemporal parameters and kinematics demonstrated the potential advantages of RAGT.

There are some limitations to this study. First, it was a small sample size study; it is possible that observations with larger sample sizes will identify more certain results. Second, with the experimental group in the process of intervention, the degree of body weight support is as the intervention process gradually reduced, so it is difficult to determine the effects of the different degrees of body weight support on RAGT; excessive body weight supports may affect peripheral information feedback, leading to difficulties of robot gait pattern input; further research should be focused on investigating RAGT effect under different degrees of body weight support. In addition, the intervention period of this study was 4 weeks, and there was no follow-up, so the long-term effects of RAGT on walking ability after stroke could not be determined. Therefore, future studies should address these limitations and recruit a large number of patients to analyze the effects of RAGT on gait dysfunction.

## 6. Conclusions

The results of this study showed that RAGT could improve physical functions and gait ability in patients with subacute stroke. 3DGA and sEMG showed that RAGT successfully improved part of spatiotemporal parameters of patients and optimized the movement mode of the affected lower limb joints during walking, which is crucial for the improvement of walking ability of subacute stroke patients in the future.

## Figures and Tables

**Figure 1:** Patient inclusion flowchart.

**Figure 2:** Lower extremity rehabilitation robot.

**Figure 3:** Placement of 3DGA markers.

**Figure 4:** Muscles of sEMG assessment.

**Figure 5:** Modeling interface for 3D gait analysis.

**Figure 6:** Interface for surface electromyography.

**Figure 7:** Comparison of the improvement in the ROM of the bilateral hip between two groups. ^∗^: *p* < 0.05; ns: *p* > 0.05.

**Figure 8:** Comparison of the improvement in the ROM of the bilateral knee between two groups. ^∗^: *p* < 0.05; ns: *p* > 0.05.

**Figure 9:** Comparison of the improvement in the ROM of the bilateral ankle between two groups. ^∗^: *p* < 0.05; ns: *p* > 0.05.

**Figure 10:** Details of cocontraction in the swing phase of the knee and ankle. ^∗^: *p* < 0.05; ns: *p* > 0.05.

**Table 1:** Baseline comparison of patients in the experimental group and the control group.

Characteristics	Experimental group (*n* = 18)	Control group (*n* = 16)	*p* value
Age (years)	56.88 ± 10.99	60.81 ± 9.61	0.337
Onset time (months)	2.50 ± 4.00	3.50 ± 3.00	0.208
Male/female	14/4	13/3	0.803
Injury site (left/right)	11/7	8/8	0.515
FMA-LE	20.69 ± 6.76	17.31 ± 6.64	0.114
FAC	3.00 ± 1.00	3.00 ± 0.00	0.087
MAS	1.00 ± 1.00	1.00 ± 1.00	0.453
Walking speed	0.26 ± 0.19	0.31 ± 0.19	0.704
Symmetry index	0.51 ± 0.19	0.60 ± 0.25	0.678
Affected stride length	0.43 ± 0.22	0.52 ± 0.18	0.523
Unaffected stride length	0.56 ± 0.20	0.47 ± 0.23	0.469
Affected hip ROM	20.17 ± 7.51	22.69 ± 10.41	0.933
Unaffected hip ROM	34.40 ± 8.15	33.50 ± 13.50	0.938
Affected knee flexion	31.95 ± 17.45	28.94 ± 14.17	0.208
Unaffected knee flexion	61.60 ± 15.25	56.90 ± 11.67	0.717
Affected ankle ROM	18.12 ± 6.13	18.84 ± 8.22	0.820
Unaffected ankle ROM	24.38 ± 8.24	23.67 ± 9.27	0.829
6MWT	91.80 ± 141.00	117.70 ± 71.41	0.523

Values denote means ± SD unless specified otherwise. The skewed distributed variables (onset time, MAS, walking speed of the experimental group, symmetry index of the experimental group, affected stride length of the experimental group, unaffected stride length of the control group, unaffected hip ROM of the experimental group, unaffected knee flexion of the experimental group, and 6MWT of the experimental group) were presented as median ± interquartile range (IQR).

**Table 2:** Baseline characteristics of the patients with sEMG.

Characteristics	Experimental group (*n* = 17)	Control group (*n* = 13)	*p* value
Age (years)	55.31 ± 11.47	60.54 ± 10.72	0.437
Onset time (months)	3.00 ± 4.00	3.00 ± 3.00	0.175
Male/female	14/3	12/1	0.355
Injury site (left/right)	7/10	7/6	0.713
FMA-LE	19.00 ± 6.29	18.69 ± 6.56	0.443
FAC	3.00 ± 1.00	3.00 ± 0.00	0.087
MAS	1.00 ± 1.00	1.00 ± 1.00	0.350
CCI knee	0.40 ± 0.11	0.38 ± 0.10	0.818
CCI ankle	0.34 ± 0.23	0.30 ± 0.17	0.691

Values denote means ± SD unless specified otherwise. The skewed distributed variables (onset time, FAC, and MAS) were presented as median ± interquartile range (IQR).

**(a):** 

	Experimental group (*n* = 18)			Control group (*n* = 16)		
	Baseline	Post	*p*	Baseline	Post	*p*
Walking speed	0.26 ± 0.19	0.54 ± 0.26	<0.001	0.31 ± 0.19	0.33 ± 0.18	0.040
Symmetry index	0.51 ± 0.19	0.84 ± 0.16	<0.001	0.59 ± 0.25	0.65 ± 0.20	0.021
Affected stride length	0.43 ± 0.22	0.71 ± 0.22	<0.001	0.52 ± 0.18	0.56 ± 0.18	0.010
Unaffected stride length	0.56 ± 0.20	0.67 ± 0.23	<0.001	0.47 ± 0.23	0.53 ± 0.19	0.393
Affected hip ROM	20.17 ± 7.51	29.57 ± 11.40	<0.001	22.69 ± 10.41	24.91 ± 10.17	0.010
Unaffected hip ROM	34.40 ± 8.15	36.26 ± 4.08	0.018	33.50 ± 13.50	36.30 ± 10.75	0.276
Affected knee flexion	31.95 ± 17.45	45.02 ± 13.67	0.001	28.94 ± 14.17	32.29 ± 14.74	0.068
Unaffected knee flexion	61.60 ± 15.25	60.05 ± 8.40	0.983	55.63 ± 12.23	55.93 ± 12.42	0.908
Affected ankle ROM	18.12 ± 6.13	24.38 ± 5.89	<0.001	18.84 ± 8.22	22.78 ± 10.07	0.023
Unaffected ankle ROM	24.38 ± 8.24	26.05 ± 15.60	0.054	23.67 ± 9.27	23.25 ± 9.05	0.793
FMA-LE	20.69 ± 6.76	23.88 ± 6.37	<0.001	17.31 ± 6.64	18.31 ± 6.42	0.008
FAC	3.00 ± 1.00	4.00 ± 1.00	0.001	3.00 ± 0.00	3.50 ± 1.00	0.002
6MWT	91.80 ± 141.00	139.15 ± 157.45	<0.001	117.70 ± 71.41	145.39 ± 73.42	0.002

**(b):** 

	sEMG experimental group (*n* = 17)			sEMG control group (*n* = 13)		
	Baseline	Post	*p*	Baseline	Post	*p*
CCI knee	0.40 ± 0.11	0.34 ± 0.14	0.042	0.38 ± 0.10	0.40 ± 0.18	0.196
CCI ankle	0.34 ± 0.23	0.30 ± 0.16	0.691	0.30 ± 0.17	0.27 ± 0.37	0.753

Values denote means ± SD unless specified otherwise. The skewed distributed variables (walking speed in baseline of the experimental group, symmetry index in the baseline of the experimental group, affected stride length in the baseline of the experimental group, unaffected stride length in the baseline of the control group, unaffected hip ROM in the baseline of the experimental group, unaffected knee flexion of the experimental group, FAC of two groups, 6MWT of the experimental group, CCI knee in post of the sEMG control group, and CCI ankle in post of the sEMG control group) were presented as median ± interquartile range (IQR).

**(a):** 

Characteristics	Experimental group (*n* = 18)	Control group (*n* = 16)	*p* value
Walking speed	0.54 ± 0.26	0.33 ± 0.18	0.025
Symmetry index	0.84 ± 0.15	0.65 ± 0.20	0.004
Affected stride length	0.71 ± 0.22	0.56 ± 0.18	0.058
Unaffected stride length	0.67 ± 0.23	0.53 ± 0.19	0.058
Affected hip ROM	29.57 ± 11.40	24.91 ± 10.17	0.032
Unaffected hip ROM	36.26 ± 4.08	36.30 ± 10.75	0.918
Affected knee flexion	45.02 ± 13.67	32.29 ± 14.74	0.001
Unaffected knee flexion	60.05 ± 8.40	55.93 ± 12.42	0.065
Affected ankle ROM	24.38 ± 5.89	22.78 ± 10.07	0.586
Unaffected ankle ROM	26.05 ± 15.60	23.25 ± 9.05	0.159
FMA-LE	23.88 ± 6.37	18.31 ± 6.42	0.010
FAC	4.00 ± 1.00	3.50 ± 1.00	0.005
6MWT	139.15 ± 157.45	145.39 ± 73.42	0.448

**(b):** 

	sEMG experimental group (*n* = 17)	sEMG control group (*n* = 13)	*p* value
CCI knee	0.34 ± 0.14	0.40 ± 0.18	0.020
CCI ankle	0.30 ± 0.16	0.27 ± 0.37	0.983

Values denote means ± SD unless specified otherwise. The skewed distributed variables (unaffected knee flexion of the experimental group, FAC of two groups, 6MWT of the experimental group, CCI knee of the sEMG control group, and CCI ankle of the sEMG control group) were presented as median ± interquartile range (IQR).

## Data Availability

All data of the study were collected in Zhejiang Rehabilitation Medical Center, China; study was conducted with approval from the Ethics Committee of the Zhejiang Rehabilitation Medical Center (ZKLL20210701).
